# Occupational Stress among Operation Room Clinicians at Ethiopian University Hospitals

**DOI:** 10.1155/2022/2077317

**Published:** 2022-07-19

**Authors:** Belayneh Yosef, Yophtahe Woldegerima Berhe, Demeke Yilkal Fentie, Amare Belete Getahun

**Affiliations:** ^1^Department of Anesthesia, Debre-Markos University, Ethiopia; ^2^Department of Anesthesia, University of Gondar, Ethiopia

## Abstract

**Background:**

The surgical operation room is a known stressor workplace. Occupational stress can cause negative impacts on the personal well-being of healthcare professionals, health services, and patient care. Since there was limited research evidence in Ethiopia and the developing world, we aimed to determine the prevalence and factors associated with occupational stress among operation room clinicians at university hospitals in Northwest Ethiopia, 2021. *Methodology*. After ethical approval was obtained, a cross-sectional census was conducted from May 10 to June 10, 2021. The United Kingdom Health and Safety Executive's Management Standards Work-Related Stress Indicator Tool was used to assess occupational stress. Data were collected from 388 operation room clinicians and analysed by using binary logistic regression analysis.

**Results:**

The prevalence of occupational stress was 78.4%. Rotating work shifts (AOR: 2.1, CI: 1.1–4.7), working more than 80 hours per week (AOR: 3.3, CI: 1.5–3.8), use of recreational substances (AOR: 2.1, CI: 1.1–3.8), being an anesthetist (AOR: 4.1, CI: 1.7–10.0), and being a nurse (AOR: 4.0, CI: 1.7–9.7) were found significantly associated with occupational stress.

**Conclusion:**

We found that there was high prevalence of occupational stress among operation room clinicians and factors associated with occupational stress were rotating work shifts, working more than 80 hours per week, use of recreational substances, being an anesthetist, and being a nurse. Hospitals are advised to arrange occupational health services for operation room clinicians, prepare sustainable training focused on occupational health, and reorganize shifts, working hours, and staffing.

## 1. Introduction

Occupational stress is a mental, emotional, and physical strain or tension which is due to an interaction between personal and professional traits. Exposure to stress conditions for a long and steady period can lead to burnout syndrome. Occupational stress results in impaired job performance, poor quality of service, and drug addiction and suicide among professionals [1–4]. In previous studies, the prevalence of occupational stress among healthcare professionals was reported in range from 32% to 92% [2, 4–15].

It was observed that anesthesiology, surgery, and surgical nursing are universally recognized as the most stressful jobs and decreased the tendency of trainees to join those stressful professions. Some of the possible reasons for high levels of stress among operation room clinicians are long working hours, inadequate sleep, fatigue and burnout, demand for interpersonal relations and team work, complexity of tasks, need for continuous vigilance, unpredictability of work and outcomes, occurrence of adverse events and complications, fear of litigation and violence, competence, and production pressures [13, 16–18]. Furthermore, the pandemic of coronavirus disease-2019 (COVID-19) has been exerting extra workload and mental instability to operation room clinicians [19–21]. The recent study by Meng et al. reported that nurse anesthetists were in danger of occupational stress and burnout and urged managers to give attention to the situation [22]. It is recommended that operation room clinicians need to be stress-free to deliver optimal care and ensure infection control [19, 23].

Occupational stress among operation room clinicians has multiple worst consequences such as depression, anxiety, poor family relationships, poor friendship, difficult relationships with colleagues, addiction to alcohol and/or drugs, marital dysfunction, divorce, premature aging, suicide, poor judgment in decision-making, decreased efficiency, medical errors, adverse events among patients including avoidable deaths, hostility towards patients, and diminished commitment, disengagement, and early retirement. All of these consequences of occupational stress have large negative impacts on the quality of healthcare and healthcare cost implications [13, 24–28]. Stress also increased the rate of dropout from training in those professions. This situation decreases the number of professionals in the field and has large negative implications for developing countries that have preexisting critical shortage of operation room clinicians. It also viciously leads to further increment of burden and stress among existing healthcare professionals [28, 29].

Despite disputing results, previous studies have reported that age, sex, marital status, rearing children, addiction, educational level, profession, working shifts and time, work experience, case load, and salary were found significantly associated with occupational stress among healthcare professionals [2, 6, 7, 9, 10, 17, 21, 25, 30–33]. Therefore, the current study aimed to determine the prevalence and factors associated with occupational stress among operation room clinicians at university hospitals in Northwest Ethiopia.

## 2. Methodology

A cross-sectional census was conducted from May 10 to June 10, 2021 at university hospitals in Northwest Ethiopia. There were only two university hospitals in the area which are University of Gondar Comprehensive Specialized Hospital (UoGCSH) and Tibebe-Ghion Specialized Hospital (TGSH). The hospitals were found in Gondar and Bahirdar cities, respectively. During the data collection period, UoGCSH had 14 operation theatres (4, general surgical; 1, orthopedic; 2, gynecologic; 2, obstetric; and 2, ophthalmic) and TGSH had 10 operation theatres (7, general surgical; 2, orthopedic; and 1, obstetric). There were a total of 480 operation room clinicians working at both universities. The UoGCSH had 274 operation room clinicians (anesthetists = 70, nurses = 65, and surgical staff = 139) and TGSH had 206 operation room clinicians (anesthetists = 24, nurses = 60, and surgical staff = 122). A total of 480 operation room clinicians at both university hospitals were approached.

All operation room clinicians working in the hospitals were included in this study and clinicians who had work experience less than 6 months and those who were on leave were excluded. The dependent variable was occupational stress and independent variables were sociodemographic and behavioral variables (age, sex, educational level, marital status, having children, salary, work experience, and addiction) and institutional variables (workload, hours, working shift, part-time employee, and permanent employment).

Occupational stress was measured by using United Kingdom Health and Safety Executive's Management Standards Work-Related Stress Indicator Tool developed by Health and Safety Executive of United Kingdom which contains 35 items. Each item was graded in Likert scale (1, never; 2, rarely; 3, sometimes; 4, often; 5, always). Participants whose stress scores were above the mean score were considered to have occupational stress. The tool was validated by a previous study [34].

Use of recreational substances: consumption of recreational substances such as alcohol, khat, cigarettes, and alike regardless of the amount and frequency of use for the past 3 months [14].

Ethical approval was obtained from Ethical Review Committee of School of Medicine, University of Gondar, before data collection in the study areas. After a brief explanation, informed consent was obtained from each study participant. Confidentiality was guaranteed by removing personal identifiers and keeping the raw data in secured areas, and data were collected through self-administered, semistructured questionnaires which included UK Health and Safety Executive's Management Standards Work-Related Stress Indicator Tool. The collected data were checked, cleaned, and analysed by using STATA version 14.1 statistical software. Distribution of the data and model fitness were checked by the Shapiro–Wilk test and Hosmer–Lemeshow test, respectively. Binary logistic regression was performed to examine the associations of independent variables with occupational stress, and the strength of associations was measured by adjusted odds ratio at 95% confidence interval. Variables with *p* value less than 0.05 were considered to have statistically significant association.

## 3. Results

Four hundred fifty operation room clinicians in 2 university hospitals in Northwest Ethiopia were approached and data from 388 (86.2%) participants were used for the final analysis. The majority of clinicians were males 306 (78.9%) and single 202 (52%). The age of the participants ranges from 23 to 51 with a median (IQR) age of 29 (27–32) years. More than half of the respondents 201 (51.8%) had an age between 25 and 29 years. Most of the operation room clinicians 249 (64.2%) had first degree and 351 (90.5%) had work experience of less than or equal to 5 years. More than two-thirds, 260 (67%) of the clinicians had reported that they were working in fixed shifts (Table 1).

Regarding the perception of operation room clinicians towards their workplace, 229 (59%) participants perceived that there was a good workplace relationship, and 228 (58.8%) participants reported that administrator/managerial support was good at their workplace. Only 81 (20.9%) clinicians had reported for role ambiguity at the workplace (Figure 1).

The overall prevalence of occupational stress among operation room clinicians was 78.4% (CI: 42%–2.5%). In the bivariate binary logistic regression analysis, age, salary, educational status, profession, type of work contract, working shifts, working time per week, and use of recreational substances were found fit to enter the final multivariate binary logistic regression analysis (*p* value <0.2). In the multivariate analysis, rotating work shift,working time per week greater than 80 hours, use ofrecreational substances, being an anesthetist, and being anurse were found significantly associated with occupational stress among operation room clinicians (*p* value <0.05).

Operation room clinicians who were working on rotating work shifts were more than twice likely to have occupational stress compared to those who were working on fixed work shifts (AOR: 2.1, CI: 1.1–4.7). The possibility to develop occupational stress was more than 3 times higher when operation room clinicians work for more than 80 hours per week than working for less than 50 hours per week (AOR: 3.3, CI: 1.5–3.8). Use of recreational substances had doubled the occurrence of occupational stress among operation room clinicians (AOR: 2.1, CI: 1.1–3.8). Anesthetists and operation room nurses were found to have occupational stress of more than 4 folds compared to the surgical staff (AOR: 4.1, CI: 1.7–10.0) and (AOR: 4.0, CI: 1.7–9.7), respectively (Table 2).

## 4. Discussion

The prevalence of occupational stress was high (78.4%) among operation room clinicians, and it is similar to a study done among nurses in Iran [10]. However, it was higher compared to studies performed by Birhanu et al. and Godifay et al. in which 68.2% and 46.9% healthcare professionals were found to have occupational stress, respectively [9, 35]. The discrepancies might be explained by the inclusion of all healthcare professionals in those studies, while our study included only operation room clinicians. The operation room is considered as one of the most stressful parts of hospitals. A study performed by Anand and Mejid found that 56.3% of nurses had occupational stress [6]. The difference might be due to the tools used to assess occupational stress as in the previous study, the nursing stress scale was used, while we used United Kingdom Health and Safety Stress Indicator Tool. Additionally, the exclusive participation of nurses in the previous study could be a possible reason for deviances. The high prevalence of occupational stress among the operation room clinicians reported in the current study may reflect understaffing, lacking adequate resources, and higher workload in the operation rooms [36]. Furthermore, working in teaching hospitals was found associated with occupational stress and explained by additional academic tasks that could increase workload such as teaching and learning programs, paper work, supervision, and advisorship [10]. In contrast, the prevalence of occupational stress in the current study was lower compared to the studies performed by Wu et al. and Bhatia et al. In the aforementioned studies, occupational stress was assessed by using different tools among female nurses who were working in larger hospitals, which are expected to have more workload [8, 37].

Working more than 80 hours per week has increased the occurrence of occupational stress by three folds compared to working less than 50 hours per week. This finding is consistent with a study conducted by Ebrahimi and Kargar [32]. Increased workload and over commitment were found associated with occupational stress and have negative impact on personal well-being, organizational performance, and patient outcome [28, 38, 39]. Working in rotating shifts was found significantly associated with occupational stress compared to working fixed shifts, and these results were supported by previous studies [7, 14].

Use of recreational substances has doubled the odds of having occupational stress. Many recreational substances have paradoxical effects that manifest as primary rewarding properties that can counterbalance or mask their stress-provoking effects [37]. Coping with stress was the leading reason among healthcare professionals for drinking alcohol. About 34% of participants responded that they used recreational substances to feel better, and 22% used substances to help them get through stressful events [38]. Similary, Mikalauskas et al. reported that the likelihood of sedative medication abuse was nearly 5 times and alcohol abuse was over 2 times among anesthetists [40].

Our study revealed that 87.0% of anesthetists were found to have occupational stress which was the highest compared to the nurses and surgical staff. The likelihood of anesthetists to be found stressed was over four times compared to the surgical staff. This finding might be explained by the anticipation of perioperative difficulties and adverse events, being challenged with complex cases, high demand of interpersonal interactions, extra load of academic activities, long working hours, high demand of continuous vigilance, unpredictability of work, poor working conditions, keeping oneself up to date with evolving science and technologies, and fear of litigation and violence [15, 16, 41]. A study performed by Birhanu et al. reported a higher prevalence of occupational stress among anesthetists compared to residents, even though it did not demonstrate statistically significant association [9]. Studies conducted by Azizpour et al. and Eskola et al. also revealed that anesthetists were more stressed than nurses [30, 42]. In contrast, a small-scale pilot study done by Kang et al. among South Korean surgeons showed that surgeons had higher occupational stress than other professionals in Korea [29].

Next to anesthetists, we found that 85.5% of operation room nurses stated occupational stress, and they are four times more likely to be found stressed compared to the surgical staff. This is comparable to a study that reported 87.4% of nurses were found stressed [8]. Supporting our finding, Hull et al. found that circulating nurses were more stressed preoperatively, eventhough assistant surgeons were more stressed intraoperatively and postoperatively [43]. High prevalence of occupational stress might arise from the physical, social, psychological, and aspects of the work environment. High prevalence of occupational stress might be explained by high case load, lack/shortage of resources for nursing practice, lack of power, role ambiguity and conflict, being undervalued, work redundancy, and unclear career development and promotion prospects. High levels of occupational stress can result in burnout and high turnover that adversely affect the health service and patient care [44]. Pačarić et al. justified the high prevalence of occupational stress among surgical nurses by financial issues, public criticism towards women, fear of litigation, and workplace organization [33]. Furthermore, the numbers of anesthetists and nurses were lower compared to the surgical staff in both hospitals. This could exert more workload on those professionals and that could end up in occupational stress.

Occupational stress is a common public health problem which can result in poor quality healthcare which is a major public health problem itself [44]. Therefore, it is mandatory to improve essential components of work climate through making operation room clinicians feel important parts of the organization, giving recognition for delivered work, encouraging development, and providing sufficient opportunities to learn and to grow [45].

This census was conducted at two university hospitals and the first of its type in the country. However, the cross-sectional design could not show tempora1 relationships. Since occupational stress is highly subjective and psychological, we recommend to future researchers to assess it by using qualitative approaches that would provide more concise and better meaningful information about occupational stress among operation room clinicians.

## 5. Conclusions

There was a high prevalence of occupational stress among operation room clinicians. Rotating work shifts, working more than 80 hours per week, use of recreational substances, being an anesthetist, and being a nurse were found significantly associated with occupational stress. The hospitals are advised to arrange occupational health counselling and support services for operation room clinicians, prepare sustainable training focused on occupational health, and reorganize shifts, working hours, and staffing.

## Figures and Tables

**Figure 1:** Perception towards workplace among operation room clinicians in UoGCSH and TGSH, Northwest Ethiopia, 2021 (*N* = 388).

**Table 1:** Sociodemographic characteristics of operation room clinicians in UoGCSH and TGSH, Northwest Ethiopia, 2021 (*N* = 388).

Variables	Categories	Frequency (*n*)	Percentage (%)
Sex	Female Male	82 306	21.1 78.9

Age	<25 25–29 30–34 ≥35	10 201 129 48	2.6 51.8 33.2 12.4

Profession	Anesthetists Nurses Surgical staff	77 121 190	19.8 31.2 49

Marital status	Single Married Divorce/widowed/separated	202 181 5	52.1 46.6 1.3

Educational status	Diploma or bachelors' degree Masters' degree and above	262 126	67.5 32.5

Work experience	≤5 years >5 years	351 37	90.5 9.5

Monthly salary (ETB)	<5000 5000–10000 >10000	24 218 146	6.2 56.2 37.6

ETB, Ethiopian birr (currency: 1 USD = 49.7 ETB).

**Table 2:** Binary logistic regression analysis: factors associated with occupational stress among operation room clinicians in UoGCSH and TGSH, Northwest Ethiopia, 2021 (*N* = 388).

Variables	Occupational stress		Odds ratio	
	No, *n* (%)	Yes, *n* (%)	COR (95% CI)	AOR (95% CI)
Age				
<25	1 (10.0)	9 (90.0)	4.1 (0.5–35.3)	2.2 (0.2–21.6)
25–29	33 (16.4)	168 (83.6)	2.3 (1.1–4.7)	1.4 (0.6–3.2)
30–34	35 (27.1)	94 (72.9)	1.2 (0.6–2.5)	0.9 (0.4–2.1)
>35	15 (31.3)	33 (68.8)	1	1

Monthly salary (ETB)				
<5000	3 (13.6)	21 (86.4)	2.6 (0.8–9.3)	1.2 (0.3–5.5)
5000–10000	41 (19.4)	177 (80.6)	1.6 (1.0–2.7)	0.8 (0.4–1.6)
>10000	40 (27.4)	106 (72.6)	1	1

Educational status				
Diploma or Bachelors' degree	47 (17.9)	215 (82.1)	1.9 (1.2–3.1)	1.3 (0.6–2.8)
Masters' degree and above	37 (29.4)	89 (70.6)	1	1

Use of recreational substance				
Yes	26 (57.8)	19 (42.2)	1.4 (0.8–2.4)	2.1 (1.1–3.8)^*∗*^
No	58 (23.8)	186 (76.2)	1	1

Profession				
Anesthetist	10 (13.0)	67 (87.0)	2.7 (1.3–5.6)	4.1 (1.7–10.0)^*∗*^
Nurses	20 (16.5)	101 (83.5)	2.0 (1.1–3.6)	4.0 (1.7–9.7)^*∗*^
Surgical staff	54 (28.4)	136 (71.6)	1	1

Working shifts				
Fixed	66 (25.3)	195 (74.7)	1	1
Rotating	18 (14.2)	109 (85.8)	1.9 (1.1–3.4)	2.1 (1.1–4.2)^*∗*^

Working hours per week				
<50	50 (26.0)	142 (74.0)	1	1
50–65	14 (22.2)	49 (77.8)	1.2 (0.6–2.4)	1.4 (0.7–2.9)
66–80	10 (18.2)	45 (81.8)	1.6 (0.7–3.4)	2.3 (0.9–5.4)
>80	10 (12.8)	68 (87.2)	2.4 (1.1–5.0)	3.3 (1.5–7.4)^*∗*^

Permanent work contract				
Yes	58 (24.2)	182 (75.8)	1	1
No	26 (17.6)	122 (82.4)	1.5 (0.9–2.3)	1.8 (0.9–3.5)

^∗^: Significant in the multivariate binary logistic regression analysis (*p*-value <0.05). AOR: adjusted odds ratio, CI: confidence interval, COR: crudes odds ratio, ETB: Ethiopian Birr (currency: 1 USD = 49.7 ETB).

## Data Availability

The data used to support this study are available from the corresponding author upon request.

## Abbreviations

AOR: Adjusted odds ratio
CI: Confidence interval
COVID-19: Coronavirus disease-2019
TGSH: Tibebe-Ghion Specialized Hospital
UoGCSH: University of Gondar Comprehensive Specialized Hospital.
